The article "Analysis of Maternal and Infant Outcomes and Related Factors of Vaginal Delivery of Second Pregnancy after Cesarean Section" was retracted in 2023. Reasons: signs of a paper mill; compromised peer review; unreliable results or conclusions.

# Analysis of Maternal and Infant Outcomes and Related Factors of Vaginal Delivery of Second Pregnancy after Cesarean Section

**DOI:** 10.1155/2022/4243174

**Published:** 2022-10-13

**Authors:** Xing Pan, Shuhui Sha, Shuxia Xu, Bingqing Zhan, Xue Guan, Fang Ling

**Affiliations:** ^1^Department of Obstetrics, Suzhou Kowloon Hospital, Shanghai Jiao Tong University School of Medicine, Suzhou, Jiangsu 215000, China; ^2^Department of Gynaecology, Suzhou Kowloon Hospital, Shanghai Jiao Tong University School of Medicine, Suzhou, Jiangsu 215000, China; ^3^Department of Nursing, Suzhou Kowloon Hospital, Shanghai Jiao Tong University School of Medicine, Suzhou, Jiangsu 215000, China

## Abstract

**Objective:**

To explore the clinical effect of different delivery methods and the safety of vaginal delivery of second pregnancy after cesarean section and analyze the related factors.

**Methods:**

A total of 738 eligible pregnant women who underwent cesarean section from September 2018 to August 2020 were randomly selected from our hospital. Among them, 527 pregnant women successfully delivered vaginally were selected as the observation group, and 211 pregnant women who failed vaginal delivery were selected as the control group. To analyze the factors that influence the success of vaginal delivery of second pregnancy after cesarean section and compare the outcomes of mother and infant in two groups.

**Results:**

There was no significant difference in age, prenatal body mass index (BMI), and thickness of lower uterine segment between the two groups (*P* > 0.05). There were significant differences in fetal head orientation, fetal abdominal circumference, fetal biparietal diameter, uterine height, premature rupture of membranes, Bishop score, and epidural anesthesia during labor between the two groups (*P* < 0.05). Multivariate logistic regression analysis showed that fetal abdominal circumference, fetal head orientation, Bishop score, and epidural anesthesia during labor were independent factors affecting the success of VBAC (*P* < 0.05). There was no significant difference in the incidence of uterine rupture between the two groups (*P* > 0.05). The amount of postpartum hemorrhage in the observation group was significantly lower than that in the control group (*P* < 0.05). There was no significant difference in Apgar score, asphyxia rate, and hospitalization rate between the two groups (*P* > 0.05). There was no significant difference in the incidence of complications between the two groups (*P* > 0.05).

**Conclusion:**

There are many factors that influence the success of vaginal delivery after cesarean section. Through prenatal comprehensive evaluation of vaginal delivery conditions, we can guide the parturient to choose a reasonable mode of delivery, reduce the incidence of complications, and improve the outcome of mother and baby.

## 1. Introduction

In recent years, with the continuous maturity and development of cesarean section, the pain experienced by mothers during delivery has been significantly reduced, and the success rate and safety of cesarean section have been significantly improved [1, 2]. However, cesarean section is the most common cause of uterine scar formation, and scar uterus is prone to uterine rupture, massive bleeding, and other adverse phenomena during the second pregnancy, which poses a serious threat to the health and life safety of mother and baby [3, 4]. In the past, cesarean section was more preferred during delivery, but with the change of medical concepts and health awareness, natural delivery was more advocated clinically [5]. Vaginal delivery has small injury on puerpera and the hospital stay is short, which is conducive to postpartum recovery. Besides, vaginal delivery is beneficial to fetus, which reduces the incidence of neonatal diseases [6]. At present, trial of labor after cesarean section (TOLAC) can reduce the overall cesarean section rate and the risk of complications of pregnancy, which is widely recognized in clinic [7, 8].

Therefore, this study selected 738 women who were pregnant again after cesarean section in our hospital as the research object, aimed at exploring the clinical effects of different delivery methods of pregnant again after cesarean section and the safety of vaginal delivery and analyze the relevant influencing factors.

## 2. Materials and Methods

### 2.1. General Information

From September 2018 to August 2020, 527 pregnant women undergoing vaginal delivery (VBAC) after cesarean section in our hospital were randomly selected as the VBAC group. Among them, the age of the enrolled was 18-42 years, the average age was 31.55 ± 3.86 years, the gestation was 31-41 weeks, the median value was 39.29 weeks (38.43, 40.00), and the interval between the last cesarean section was 1-16 years, including 7 cases in 1-2 years, 198 cases in 2-5 years, 258 cases in 5-10 years, and 64 cases in more than 10 years.

A total of 211 pregnant women with failed vaginal delivery (VBNC) after cesarean section at the same period were selected as the VBNC group. They were 21-48 years old, with an average age of 31.36 + 4.56 years, 32 + 2 − 41 + 3 weeks pregnant, with a median value of 39.36 weeks (38.43, 40.03). The time from the last vaginal delivery was 1-16 years, including 38 cases in 1-2 years, 103 cases in 2-5 years, 54 cases in 5-10 years, and 16 cases in more than 10 years. This study was approved by the Ethics Committee of Suzhou Kowloon Hospital, Shanghai Jiao Tong University School of Medicine.

Inclusion criteria: (1) the pregnant women who became pregnant again after cesarean section met the relevant diagnostic criteria after cesarean section, and all had one cesarean section experience; (2) the time from the second pregnancy to the previous cesarean section was >2 years, and all of them were singleton cephalic; (3) patients and their families should be informed and sign informed consent.

Exclusion criteria: (1) prenatal B-ultrasound showed pelvic abnormalities, scar position, and uterine thickness <0.2 cm; (2) there were complications such as incision infection and postpartum hemorrhage after the previous cesarean section; (3) complicated with pregnancy diabetes, pregnancy induced hypertension, and other diseases; (4) complicated with severe cognitive impairment and unable to cooperate with treatment.

### 2.2. Pregnancy Management

TOLAC pregnant women receive the whole process management of pregnancy, nutrition, and exercise guidance during pregnancy, and they control their body mass during pregnancy. In the third trimester of pregnancy, the thickness and continuity of the myometrium at the incision of the uterus were evaluated by ultrasound, the weight of the fetus was evaluated, and the pelvic condition was measured. At least two doctors with the title of deputy director were evaluated to make a delivery plan.

### 2.3. Production Process Management

If there was no indication of induction of labor, pregnant women expect natural labor; those who met the indications for induction of labor were admitted to the hospital for induction of labor. According to the cervical score, small doses of oxytocin were selected for intravenous drip induction of labor, or water capsules were used to promote cervical maturation. During VBAC, continuous fetal heart rate monitoring should be carried out, and preparations for cesarean section should be made. In case of maternal and infant abnormalities, the surgical indications should be relaxed and emergency cesarean section should be carried out.

### 2.4. Analysis of Relevant Factors

The possible factors affecting the success of VBAC were recorded, including age, prenatal BMI, fetal abdominal circumference, fetal biparietal diameter, premature rupture of membranes, Bishop score, uterine height, fetal head orientation, thickness of lower uterine segment, and epidural anesthesia during labor.

### 2.5. Observation Index

1. Bishop scoring standard [9] including 5 items such as cervical dilatation, disappearance of cervical canal, fetal presentation position, cervical orifice position, and cervical stiffness, the total score of cervical maturity was ≥6 points
2. Apgar score, neonatal asphyxia rate, and neonatal hospitalization rate of the two groups were statistically analyzed. The Apgar score is based on a total score of 1 to 10. The higher the score, the better the baby was doing after birth. A score of 7, 8, or 9 was normal and was a sign that the newborn was in good health
3. The incidence of uterine rupture in the two groups was counted, and the bleeding volume at 2 and 24 hours after delivery was recorded
4. The incidence of pregnancy complications in two groups were recorded, including GDM, hypoactive hypothyroidism, thyroid hyperactivity, syphilis, gestational hypertension, and liver injury

### 2.6. Statistical Analysis

The data of this study were processed and analyzed in the software SPSS 20.0. The measurement data generated in the study were described in the form of mean ± mean and parallel *t*-test was performed. The count data in the study were expressed by percentage [*n* (%)]. *X*^2^ test was used. Set the statistical test level as: *α* = 0.05, *P* < 0.05 was statistically significant. The relative risk or value and 95% confidence interval (95% CI) were calculated for various factors. After multivariate logistic analysis, *P* < 0.05 was considered as statistically significant.

## 3. Results

### 3.1. Comparison of the Results of Vaginal Trial Labor

A total of 738 women who became pregnant again after cesarean section underwent vaginal trial delivery, and 527 women delivered vaginally, accounting for 71.41%. 211 cases of failed trial delivery were changed to cesarean section, 47 cases of parturients gave up continuing trial delivery, 32 cases of continuous pain in the lower abdomen, 63 cases of fetal head descent stagnation, 53 cases of active early stagnation, and 16 cases of cervical edema.

### 3.2. Comparison of Related Factors Affecting the Success of VBAC

There was no significant difference in age, prenatal body mass index (BMI), and thickness of lower uterine segment between the two groups (*P* > 0.05); There were significant differences in fetal head orientation, fetal abdominal circumference, fetal biparietal diameter, uterine height, premature rupture of membranes, Bishop score, and epidural anesthesia during labor between the two groups (*P* < 0.05), as shown in Table 1.

### 3.3. Multivariate Logistic Regression Analysis

The results of multivariate logistic regression analysis showed that fetal abdominal circumference, fetal head orientation, Bishop score, and epidural anesthesia during labor were the independent factors affecting the success of VBAC (*P* < 0.05), as shown in Table 2.

### 3.4. Comparison of Delivery between Two Groups

There was no significant difference in the incidence of uterine rupture between the two groups (*P* > 0.05). The amount of postpartum hemorrhage in the VBAC group was significantly lower than that in the VBNC group at 2, 12, and 24 hours (*P* < 0.05), as shown in Figure 1.

### 3.5. Comparison of Newborns in Two Groups

There was no significant difference in Apgar score, asphyxia rate, and hospitalization rate between the two groups (*P* > 0.05), as shown in Figure 2.

### 3.6. Comparison of Pregnancy Complications

By comparing the complications of pregnant women during pregnancy, it was found that there were more pregnant women with gestational diabetes mellitus (GDM) in the two groups. The data showed that the highest incidence of pregnancy complications was pregnancy diabetes, and the incidence of VBAC group (22 cases) was higher than that of VBNC group (14 cases). But there was no significant difference in the incidence of complications between the two groups (*P* > 0.05). In the absence of obvious contraindications to delivery, vaginal delivery could be performed under close monitoring. As shown in Figure 3.

## 4. Discussion

In recent years, the clinical cesarean section rate in China has been rising, the research on cesarean section has been increasing, and the severity of re pregnancy after cesarean section is getting higher and higher. The common clinical indications of cesarean section include ectopic placenta, fetal distress, cephalopelvic disproportion, and maternal fear of vaginal delivery pain. Some obstetricians have the misconception that “one cesarean section, all cesarean sections in the future”. It is reported in the literature that vaginal trial delivery after cesarean section can lead to uterine rupture and neonatal asphyxia. Failure of vaginal trial delivery will increase postpartum hemorrhage. In serious cases, the uterus will be removed. Most mothers will choose cesarean section again [10]. In addition, the doctor-patient relationship is tense, and pregnant women are unwilling to bear the risk of vaginal trial of pregnancy after cesarean section, which greatly increases the cesarean section rate. However, due to the influence of the previous cesarean section, there are different degrees of adhesion in the abdominal cavity. The second cesarean section may cause uterine tissue damage and increase the amount of postpartum hemorrhage. In 2010, the American Association of Obstetricians and Gynecologists formulated the VBAC guideline [11]. In 2010, the American Association of Obstetricians and Gynecologists formulated the VBAC guideline.

The results of this study showed that 738 pregnant women who were pregnant again after cesarean section performed vaginal trial delivery, and the natural delivery rate was 71.41% (527/738), which was equivalent to 60%~80% reported at home and abroad [11, 12], which may be related to the improvement of the educational level of the mothers and their families and the improvement of their understanding of the advantages and disadvantages of cesarean section. In addition, 28.59% of the patients who transferred to cesarean section may have insufficient understanding of cesarean section, and even had feudal ideas, hoping to give birth in “auspicious time”. Moreover, the pregnant women lack confidence in the trial birth, give up halfway, and eventually change to cesarean section, which is also the reason for the high cesarean section rate. Some studies have shown that [13], maternal age and BMI last year are the factors affecting VBAC. Obese pregnant women have excessive uterine enlargement and primary uterine atony, which leads to poor labor force in the second stage of labor and abnormal labor process. Foreign studies have shown that, taking the age of pregnant women as the boundary, the success rate of vaginal trial birth under 40 years old is higher than that over 40 years old. The results of this study showed that maternal age and preoperative BMI had no significant impact on pregnancy and vaginal delivery after cesarean section (*P* > 0.05). It was speculated that there were more cases with good lifestyle and moderate body weight. In addition, the overall childbearing age of maternal was small, which may also be related to the small number of included samples. Fetal abdominal circumference, fetal biparietal diameter, and uterine height are common indicators to determine fetal body mass. The heavier the fetus, the lower the success rate of vaginal delivery [14]. A study showed that [15], uterine height, fetal abdominal circumference, and fetal biparietal diameter are the factors that affect the success of transvaginal delivery of second pregnancy after cesarean section. Previous studies have shown that [16], fetal factors include macrosomia, twins, fetal abnormalities, and fetal distress, which make mothers choose cesarean section to end delivery.

This study showed that there was a significant difference of Bishop scores between the two groups (*P* < 0.05). Bishop score is an important indicator to evaluate cervical maturity, including cervical orifice position, cervical tube regression, cervical hardness, cervical orifice expansion degree, and the position of presentation. The higher the Bishop score, the higher the degree of cervix, and the higher the success rate of induction of labor [17]. Some studies have shown that cervical dilatation <4 cm and the first exposure position >2 cm will increase the failure rate of trial delivery. Previous studies have shown that [18], Bishop scores can predict the success of cesarean section, pregnancy again, and vaginal delivery to a certain extent. In the process of delivery, the orientation of the fetal head is very important. Occipital posterior position and occipital transverse position can make the maternal pain unbearable in the active period, cervical edema, irritability, abnormal labor process, etc., which will reduce the success rate of trial labor, and at the same time, they will press the lower part of the uterus for a long time, increasing the incidence of uterine rupture. Some literature studies have shown that [19], the higher the thickness of the lower uterine myometrium, the higher the success rate of vaginal delivery in another pregnancy. If the thickness of the lower segment of the uterus is >3 mm, the risk of uterine rupture due to scar tearing in the last operation is small, which significantly improves the success rate of vaginal delivery [20]. The results of this study showed that there was no significant difference in the thickness of the lower uterine segment between the two groups (*P* > 0.05), which was presumably related to the strict screening of the included samples. Studies have shown that [21], mothers choose cesarean section because they fear the pain of natural childbirth. With the development of medicine, painless delivery is widely used in clinic. Epidural anesthesia can effectively reduce labor pain and improve the rate of natural delivery. A study showed that [22], continuous epidural anesthesia used for painless delivery can shorten the second stage of labor, reduce the cesarean section rate, and have very little impact on mother and baby. A study found that epidural anesthesia can reduce the stress response caused by labor pain and ensure the smooth progress of natural labor [23]. It is currently believed that epidural anesthesia during labor can effectively alleviate pain, will not increase the failure rate of VBAC, and will not mask the symptoms and signs of uterine rupture. In 527 cases of successful vaginal delivery, the use rate of epidural anesthesia was 92.22%. It can be seen that epidural anesthesia during labor is conducive to improving the success rate of VBAC. In recent years, with the continuous development of clinical anesthesia technology in China, a large number of anesthesia technologies have been applied to labor analgesia. Epidural intermittent pulse injection technology can delay the time of the first PCA, reduce the dosage of narcotic drugs, shorten the second stage of labor, and reduce the rate of dystocia. Previous studies have shown that epidural intermittent pulse injection technology can be safely and effectively applied to painless delivery, reducing the incidence of nausea and vomiting, skin itching, motor block, lower limb numbness, and improving maternal satisfaction [24].

In addition to the amount of postpartum hemorrhage, there was no significant difference between the two groups in maternal and infant outcomes, especially in the rate of uterine rupture, Apgar score of newborns, asphyxia rate, and hospitalization rate (*P* > 0.05), indicating that vaginal delivery of pregnancy after cesarean section was safe and reliable for both mothers and infants when conditions permit. Some studies believe that pregnant women who become pregnant again after cesarean section should make prenatal preparations and strictly grasp the indications of vaginal delivery, which can improve the rate of vaginal delivery [25]. Most studies have shown that VBAC can improve the perinatal condition, has no adverse effect on newborns, and has high safety. It can be seen that the success of vaginal trial delivery after cesarean section is undoubtedly the best mode of delivery. Of course, in the prenatal period, senior doctors should evaluate the risk of vaginal trial birth, determine the people suitable for vaginal trial birth, patiently explain the advantages and disadvantages of cesarean section and natural delivery in detail, help mothers build confidence, and introduce the advantages and disadvantages of painless delivery with epidural anesthesia. From the domestic and foreign research results, clinical application results, and other aspects, we can help mothers scientifically choose analgesic methods and effectively alleviate the pain of childbirth, so as to reduce the complications caused by blind delivery and improve the success rate of VBAC [25, 26].

There are some limitations in our study. First, the sample of our study was relatively small. Second, our study had regionalism, which could not represent the whole pregnant women. Therefore, further relative studies should be carried to in the future.

To sum up, there are many factors that affect the success of vaginal delivery after cesarean section. Prenatal comprehensive evaluation of vaginal delivery conditions can guide mothers to choose a reasonable mode of delivery, reduce the incidence of complications, and improve the outcome of mother and baby.

## Figures and Tables

**Figure 1:** Comparison of delivery between two groups. Note: ^∗^*P* < 0.05, compared with the VBNC group.

**Figure 2:** Analysis of newborns in 2 groups.

**Figure 3:** Comparison of pregnancy complications.

**Table 1:** Analysis of relevant factors affecting the success of VBAC.

Factors		VBAC (*n* = 527)	VBNC (*n* = 211)
Age/years		31.55 ± 3.86	31.36 ± 4.56
Antenatal BMI/(kg/m^2^)	18.5~25	248 (47.06)	101 (47.87)
	26~30	22 (4.24)	5 (2.37)
	> 30	257 (48.76)	105 (49.76)
Fetal abdominal circumference/mm	31~34	375 (71.16)^∗^	68 (32.23)
	35~36	152 (28.84)^∗^	143 (67.77)
Biparietal diameter of fetus/cm	87~94	457 (86.72)^∗^	126 (59.72)
	95~97	98 (13.28)^∗^	85 (40.28)
Palace height/cm	32~34	492 (93.36)^∗^	89 (42.18)
	35~38	35 (6.64)^∗^	122 (57.82)
Premature rupture of membranes	Yes	339 (64.32)^∗^	42 (19.91)
	No	188 (35.68)^∗^	169 (80.09)
Bishop scores	< 6	98 (13.28)^∗^	181 (59.72)
	≥ 6	492 (93.36)^∗^	85 (40.28)
Tire head orientation	Occipital anterior position	353 (66.97)^∗^	53 (25.12)
	Occipital transverse position	116 (22.02)^∗^	53 (25.12)
	Occipital posterior position	58 (11.01)^∗^	105 (49.76)
Thickness of lower uterine segment/cm		3.20 ± 0.45	3.16 ± 0.42
Epidural anesthesia during labor	Yes	486 (92.22)^∗^	64 (30.33)
	No	41 (7.78)^∗^	147 (69.67)

Note: ^∗^*P* < 0.05, compared with the VBNC group.

**Table 2:** Multivariate logistic regression analysis.

Factors	Standard error	Partial regression coefficient	OR	95% CI	*P*
Fetal abdominal circumference	0.340	2.124	4.154	1.154~6.160	0.005
Bishop scores	0.955	3.123	7.135	1.327~4.230	0.003
Tire head orientation	0.624	3.293	7.124	1.620~6.531	0.000
Epidural anesthesia during labor	0.318	0.836	2.668	1.320~5.212	0.002

## Data Availability

Original data included/analyzed in this study are available from the corresponding author under reasonable requests.
